The article "Causes of Cancer in the World: Comparative Risk Assessment of Nine Behavioral and Environmental Risk Factors" was retracted in 2024. Reasons: plagiarism; plagiarized images; overlap with other authors' work.

# Causes of Cancer in the World: Comparative Risk Assessment of Nine Behavioral and Environmental Risk Factors

**DOI:** 10.7759/cureus.28875

**Published:** 2022-09-07

**Authors:** Khizer K Ansari, Asha Jha

**Affiliations:** 1 Pharmacology, Jawaharlal Nehru Medical College, Datta Meghe Institute of Medical Sciences, Wardha, IND

**Keywords:** cancer, deaths, site-specific, reports, paf, risk factor, causes

## Abstract

Some malignancies have very few technologies available for screening, and advancements in cancer therapy have not been as effective in lowering death as those for other chronic diseases. The major method for decreasing cancer incidence is primary avoidance through dietary and environmental changes. The potentially reversible risk factors were projected to be responsible for cancer-related mortality worldwide. Of these fatalities, many of the cases occurred in high-income nations, whereas very few cases did so in low- and middle-income countries. Risk factors in Europe and Central Asia were responsible for the majority of cancer mortality in low- and middle-income regions. Smoking, drinking alcohol, and eating few fruits and vegetables were some of the primary factors that contributed to cancer mortality both globally and in low- and middle-income countries. In high-income countries, alcohol consumption, smoking, and obesity were the main cancer-causing factors. The sexual transmission of the human papillomavirus is one of the leading risk factors for cervical cancer in women in low- and middle-income countries.

## Introduction and background

Mortality rates from all malignancies decreased by 32% globally between 1991 and 2019 in both men and women. This decrease was smaller than the drop in cardiovascular disease death rates, which fell by 9% and 14% in males aged between 30 and 69 and more than 70 and by 15% and 11% in women of similar age ranges, respectively [1,2].

Changes in risk factor exposure and the accessibility of screening instruments and medical care aﬀect mortality rates from chronic diseases in particular age groups. The death rate from cardiovascular illnesses has decreased throughout the recent decades, at least in industrialized countries, because of advancements in primary and secondary prevention and treatment [3]. However, the majority of therapeutic approaches have had less eﬀectiveness in lowering cancer-related fatalities. For instance, age-adjusted mortality rates for malignancies combined in the United States decreased modestly. Lung, prostate, and colorectal cancer death rates declined, which has led to a remarkable decline in total cancer mortality in males. The 1990s saw a rise in lung cancer mortality among women but a decrease in breast and colorectal cancer death rates. Reduced incidence was mainly to blame for reducing lung cancer mortality among males [4], likely the outcome of a reduction in smoking. The actual reason for the drop in prostate cancer mortality is unknown, and incidence rates across time may not be comparable due to advancements in diagnostic techniques and death certification [5]. Earlier diagnosis and excision of precancerous polyps, early tumor discovery, and successful therapy may be responsible for decreased death rates in colorectal cancer [6]. Increased mammography screening coverage for women with breast cancer [7] and eﬀective tamoxifen treatment and multi-agent chemotherapy have successfully decreased mortality [8]. Some diseases in adolescents and young adults, such as testicular cancer and leukemia, have also responded well to treatment [9,10]. However, the five-year survival rates for esophagus, liver, lung, stomach, and pancreatic cancers remain relatively poor (all <25%) [9].

The article "Causes of Cancer in the World: Comparative Risk Assessment of Nine Behavioral and Environmental Risk Factors" was retracted in 2024. Reasons: plagiarism; plagiarized images; overlap with other authors' work.

Even in industrialized nations, the impact of treatment on community patterns in cancer mortality is constrained by the availability of therapeutic medicines for other malignancies and access and usage constraints. While combining screening and therapy is improving at lowering cancer-related mortality, this is still the case. Therefore, primary prevention by changes in lifestyle and environment may be the most excellent alternative for reducing the heavy and rising burden of malignancies globally. It is necessary to conduct accurate and comparative evaluations of the impact of cancer risk components at the community level to develop programs and policies to carry out such interventions.

The World Cancer Report summarizes several publications that have measured the impacts of the risk factors on cancer incidence and death [11]. However, most research is limited to a single risk component, cancer location, or demographic [12-18]. According to Pisani et al. [19], roughly 16% of cancer cases globally are assumed to be caused by certain infectious organisms. Parkin et al. [20] created assignable fractions for various risk component cancer site combinations based on the study of published data. The objective of this review is to determine regional and worldwide cancer-related death rates that may be attributable to diﬀerent risk factors both individually and collectively.

## Review

Methodology

Assessed Risk Factors

To control the cumulative impact of risk variables on cancer deaths, in addition to meta-analyses and comprehensive reviews of the literature on risk components, exposure, and comparative risk conducted as part of the relative risk assessment project [21,22], we also gathered statistics from some of the new sources, as shown in Table 1 [23-31]. The following criteria were used to select the risk factors: high probability of causation; rationally complete information on community exposure and threat stages; suitable methods for extrapolation when necessary; the likelihood of being a significant contributor to the global or regional disease load; not being too specific or broad for a comparable explanation; and analysis of exposure in different populations.

The article "Causes of Cancer in the World: Comparative Risk Assessment of Nine Behavioral and Environmental Risk Factors" was retracted in 2024. Reasons: plagiarism; plagiarized images; overlap with other authors' work.

**Table 1:** Cancer risk factors, exposure variables, theoretical-minimum-risk exposure distributions, and disease outcomes.

	Exposure variable	Theoretical-minimum-risk exposure distribution	Cancer sites affected (age groups assessed)
Diet and physical inactivity			
Overweight and obesity	BMI (kg/m^2^)	21 SD 1 kg/m^2^	Corpus uteri cancer, colorectal cancers (≥30 years), post-menopausal breast cancer (45 years), gallbladder cancer, kidney cancer
Low fruit and vegetable intake	Fruit and vegetable intake per day	600 SD 50 g intake per day for adults	Colorectal cancer, stomach cancer, lung cancer, esophageal cancer (>15 years)
Physical inactivity	Three categories: inactive, insufficiently active (<2.5 hours per week of moderate-intensity activity, or <4,000 KJ per week), and sufficiently active. Activity in spare time, work, and transport considered	>2.5 hours per week of moderate-intensity activity or equivalent (4,000 KJ per week)	Breast cancer, colorectal cancer(>15 years), prostate cancer
Addictive substance			
Smoking	Current levels of smoking impact ratio (indirect indicator of accumulated smoking risk based on excess lung cancer mortality)	No smoking	Lung cancer, mouth and oropharynx cancer, esophageal cancer, stomach cancer, liver cancer, pancreatic cancer, cervix uteri cancer, bladder cancer, leukemia (>30 years)
Alcohol use	Current alcohol consumption volumes and patterns	No alcohol use	Liver cancer, mouth and oropharynx cancer, breast cancer, esophageal cancer, selected other cancers (≥15 years)
Sexual and reproductive health			
Unsafe sex	Sex with an infected partner without any measures to prevent infection	No safe sex	Cervix uteri cancer (all ages)
Environmental risks			
Urban air pollution	Estimated yearly average particulate matter concentration for particles with aerodynamic diameters <2.5 µ or 10 µ (PM2.5 or PM10)	7.5 µg/m^3^ for PM2.5, 15 µg/m^3^ for PM10	Lung cancer (>30 years)
Indoor smoke from household use of solid fuels	Household use of solid fuels	No household solid fuels use with limited ventilation	Lung cancer (coal) (>30 years)
Other selected risks			
Contaminated injections in healthcare settings	Exposure to ≥1 contaminated injection (contamination refers to potential transmission of hepatitis B virus and hepatitis C virus)	No contaminated injections	Liver cancer (all ages)

Procedures

An expert working committee evaluated published studies and additional sources in depth and methodically to obtain data about risk component disclosure and relative risk for each factor (R.R.). Additionally, the groups collected primary data, reanalyzed primary data sources, and conducted epidemiological investigations of meta-analyses. References listed in Table 1 include information on the data sources and analysis used to determine each risk factor.

The article "Causes of Cancer in the World: Comparative Risk Assessment of Nine Behavioral and Environmental Risk Factors" was retracted in 2024. Reasons: plagiarism; plagiarized images; overlap with other authors' work.

Analytical Statistics

We used the equation given in the panel or its discrete counterparts for hazard elements and express publicity information to determine the attributable populace fractions (PAF) for certain hazard factors. We calculated the proportional lower in particular site cancer mortality that might increase if exposure to every risk had been reduced to the counterfactual distribution using PAF for every danger element and most cancers webpage. The theoretical-minimum-chance publicity distribution is the publicity distribution that can bring about the lowest population threat which was used in this observation because of the counterfactual (opportunity) situation (Table 1). This method may quantify all risk variables’ potential reduction in cancer burden. The hypothetical lowest-risk exposure distribution equals zero and would reflect the least risk when it comes to risk variables for which zero exposure might be established. Zero exposure is not an acceptable option for some risk variables due to biological impossibility or lower physical exposure reduction restrictions. In an epidemiological study, we used the lowest values of these risk factors identified in certain groups. We decided on a counterfactual exposure distribution for danger variables having protective eﬀects primarily depends on a mixture of degrees seen in a high diet intake community and the level up to which health advantages may arise.

Because most cancers are due to many threat factors, PAFs for several threat components for the equal cancer region may overlap and account for more than 100%. For instance, solid fuels (coal and biomass) are used in more than 70% of Chinese households for heating and cooking [30] while >60% of Chinese males smoke. By giving up smoking or avoiding exposure to indoor coal smoke, which raises the risk of lung cancer [13], some lung cancer fatalities can be avoided. Both risk factors would be implicated in such circumstances. Due to multi-causality, many interventions can be used to prevent ailment, with the precise mix depending on expenses, the accessibility of new technology, the state of the infrastructure, and personal choices. As detailed above, we also computed the PAFs for numerous risk variables [32].

The article "Causes of Cancer in the World: Comparative Risk Assessment of Nine Behavioral and Environmental Risk Factors" was retracted in 2024. Reasons: plagiarism; plagiarized images; overlap with other authors' work.

We calculated all individual and combined PAFs after dividing the population into eight age groups. We extended the PAF by the overall local website-particular cancer deaths for the year 2001 (from WHO databases) for each global financial institution, place, age, sex, and cancer website to decide the wide variety of website-particular most cancers deaths that may be without delay attributed to a hazard element or group of hazard factors. For presentation, fatalities that might be attributed have been combined into three age categories.

Role of the Funding Source

The funding of the study had no bearing on the design, assembly, analysis, explanation, or writing of the research report. Whether to submit the survey for publication rested solely with the corresponding author who had complete access to the study’s data.

Outcome measures

Table 2 [28] shows the expected person and combined distribution of the chosen risk components to deaths for each cancer page for the global average and for each of the high- and low-income nations separately. The total effects by location for middle- and low-income countries are further categorized in Figure 1. They are categorized by sex and wealth in Figure 2 and by age in Table 3. The interactions of the nine risk components listed in Table 1 contributed to an estimated 243 million (35%) of the 7 million cancer-related deaths globally in 2001.

**Table 2:** Individual and joint contributions of risk factors to mortality from site-specific cancers.

	Total deaths	PAF (%) and number of attributable cancer deaths (thousands) for individual risk factors																	P.A.F. due to joint hazards of risks factors
World		Alcohol use	Smoking		Low fruit and vegetable intake		Overweight and obesity		Physical inactivity		Contaminated injections in healthcare settings		Indoor smoke from household use of solid fuels			Unsafe sex		Urban air pollution	
Mouth and oropharynx cancer	311,633	(16%, 51)	(42%, 131)		-		-		-		-		-			-		-	52%
Esophageal cancer	437,511	(26%, 116)	(42%, 184)		(18%, 80)		-		-		-		-			-		-	62%
Stomach cancer	841,693	-	(13%, 111)		(18%, 147)		-		-		-		-			-		-	28%
Colon and rectum cancer	613,740	-	-		(2%, 12)		(11%, 69)		(15%, 90)		-		-			-		-	13%
Liver cancer	606,441	(25%, 150)	(14%, 85)		-		-		-		(18%, 111)		-			-		-	47%
Pancreatic cancer	226,981	-	(22%, 50)		-		-		-		-		-			-		-	22%
Trachea, bronchus, and lung cancer	122,6981	-	(70%, 856)		(11%, 135)		-		-		-		(1%, 16)			-		(5 %, 64)	74%
Breast cancer	472,424	(5%, 26)	-		-		(9%, 43)		(10%, 45)		-		-			-		-	21%
Cervix uteri cancer	234,728	-	(2%, 6)		-		-		-		-		-			(100%, 235)		-	100%
Corpus uteri Cancer	70,881	-	-		-		(40%, 28)		-		-		-			-		-	42%
Bladder cancer	175,318	-	(28%, 48)		-		-		-		-		-		-			-	28%
Leukemia	263,169	-	(9%, 23)		-		-		-		-		-		-			-	9%
Selected other cancers	145,802	(6%, 8)	-		-		-		-		-		-		-			-	6%
All other countries	1,391,507	None of the selected risk factors																	0%
All cancer	7,018,402	(5%, 351)	(21%, 1493)	(5%, 374)		(2%, 139)		(2%, 135)		(2%, 111)		(<0–5%, 16)		(3%, 235)			(1%, 64)		35%
Low- and middle-income countries																			
Mouth and oropharynx cancer	271,074	(14%, 38)	(37%, 100)		-		-		-		-		-		-			-	48%
Esophageal cancer	379,760	(24%, 92)	(37%, 141),		(19%, 73)		-		-		-		-		-			-	58%
Stomach cancer	695,426	-	(11%, 74)		(19%, 130)		-		-		-		-		-			-	27%
Colon and rectum cancer	356,949	-	-		(2%, 9)		(9%, 32)		(15%, 54)		-		-		-			-	11%
Liver cancer	504,407	(23%, 117)	(11%, 56)		-		-		-		(23%, 117),		-		-			-	45%
Pancreatic cancer	116,827	-	(15%, 18)		-		-		-		-		-		-			-	15%
Trachea, bronchus, and lung cancer	770,938	-	(60%, 466)		(13%, 98)		-		-		-		(2%, 16)		-			(7%, 52)	66%
Breast cancer	317,195	(4%, 12)	-		(7%, 23)		(10%, 30)		-		-		-		-			-	18%
Cervix uteri cancer	218,064	-	(2%,4)		-		-		-		-		-		(100%, 218)			-	100%
Corpus uteri cancer	43,926	-	-		-		(37%, 16)		-		-		-		-			-	37%
Bladder cancer	116,682	-	(21%, 24)		-		-		-		-		-		-			-	21%
Leukemia	190,059	-	(6%, 11)		-		-		-		-		-		-			-	6%
Selected other cancers	88,706	(4%, 3)	-		-		-		-		-		-		-			-	4%
All other countries	882,001	None of the selected risk factors																	0%
All cancer	4,952,014	(5%, 262)	(18%, 896)	(6%, 311)		(1%, 71)		(2%, 84)		(<0-5%, 16)		(2%, 108)		(4%, 218)			(1%, 52)		34%
High-income countries																			
Mouth and oropharynx cancer	40,559	(33%, 14)	(71%, 29)		-		-		-		-		-		-			-	80%
Esophageal cancer	57,752	(41%, 24)	(71%, 41)		(12%, 7)		-		-		-		-		-			-	85%
Stomach cancer	146,267	-	(25%, 36)		(12%, 17)		-		-		-		-		-			-	34%
Colon and rectum cancer	256,791	-	-		(1%, 3)		(14%, 37)		(14%, 36 )		-		-		-			-	15%
Liver cancer	102,033	(32%, 33)	(29%, 29)		-		-		-		(3%, 3)		-		-			-	52%
Pancreatic cancer	110,154	-	(30%, 33)		-		-		-		-		-		-			-	30%
Trachea, bronchus, and lung cancer	4,556,636	-	(86%, 391)		(8%, 36)		-		-		-		(0%)		-			(3%, 12)	87%
Breast cancer	155,230	(9%, 14)	-		-		(13%, 20)		(9%, 15)		-		-		-			-	27%
Cervix uteri cancer	16,663	-	(11%, 2)		-		-		-		-		-		(100%, 17)			-	100%
Corpus uteri cancer	26,955	-	-		-		(43%, 12)		-		-		-		-			-	43%
Bladder cancer	58,636	-	(41%, 24)		-		-		-		-		-		-			-	17%
Leukemia	73,110	-	(17%, 12)		-		-		-		-		-		-			-	8%
Selected other countries	57,095	(8%, 5)	-		-		-		-		-		-		-			-	0%
All other cancers	509,507	None of the selected risk factors																	5%
All cancers	2,066,388	(4%, 88)	(29%, 596)	(3%, 64)		(3%, 69)		(2%, 51)		(<0.5%, 3)		(0%, 0)		(1%, 17)			(1%, 12)		37%

The article "Causes of Cancer in the World: Comparative Risk Assessment of Nine Behavioral and Environmental Risk Factors" was retracted in 2024. Reasons: plagiarism; plagiarized images; overlap with other authors' work.

**Figure 1:** Deaths from site-specific cancers attributable to selected risk factors in low- and middle-income countries by region. For every cancer site, solid blocks of color represent deaths not attributable to risks assessed, and broken blocks of color represent deaths attributable to selected risk factors listed in Table 1 [28].

**Figure 2:** Worldwide deaths from site-specific cancers attributable to selected risk factors by sex. For every cancer site, solid blocks of color represent deaths not attributable to risks assessed, and broken blocks of color represent deaths attributable to selected risk factors in Table 1 [28].

**Table 3:** Total cancer deaths (in thousands) by age and cancer site.

	Age			Total attributable deaths
	0–29 years	30–69 years	>70 years	
World				
Mouth and oropharynx cancer	6	204	101	163
Esophageal cancer	2	264	172	271
Stomach cancer	9	455	378	240
Colon and rectum cancer	6	282	326	79
Liver cancer	16	394	196	283
Pancreatic cancer	0.7	111	115	50
Trachea, bronchus, and lung cancer	5	684	537	908
Breast cancer	2	305	165	98
Cervix uteri cancer	11	156	67	235
Corpus uteri cancer	0.4	35	36	28
Bladder cancer	1	67	106	48
Leukemia	75	107	81	23
All cancers	122	3,783	3,013	2,427
Low- and middle-income countries				
Mouth and oropharynx cancer	6	180	85	131
Esophageal cancer	2	235	143	222
Stomach cancer	8	399	288	191
Colon and rectum cancer	6	193	158	40
Liver cancer	16	346	142	229
Pancreatic cancer	0.6	68	48	18
Trachea, bronchus, and lung cancer	4	482	284	512
Breast cancer	2	227	89	56
Cervix uteri cancer	11	146	61	218
Corpus uteri cancer	0.4	25	19	16
Bladder cancer	1	53	62	24
Leukemia	70	81	39	11
All cancers	206	2,946	1,800	1,668
High-income countries				
Mouth and oropharynx cancer	0.2	24	16	32
Esophageal cancer	0.1	29	29	49
Stomach cancer	0.5	56	90	49
Colon and rectum cancer	0.5	88	168	40
Liver cancer	0.4	48	54	53
Pancreatic cancer	0.1	43	67	33
Trachea, bronchus, and lung cancer	0.3	202	253	396
Breast cancer	0.3	79	76	42
Cervix uteri cancer	0.2	10	6	17
Corpus uteri cancer	0	10	17	12
Bladder cancer	0	14	44	24
Leukemia	4	26	43	12
All cancers	16	837	1,212	759

Cervix-uterine, lung, and esophageal cancer had the highest percentages of cancers (>60%) which may be attributed to these factors. Smoking, alcohol use, a poor diet of fruits and vegetables, and sexual transmission of HPV that results in chronic infection of oncogenic viruses were the greatest risk factors for these malignancies. The malignancies with the lowest cumulative PAFs, leukemia (9%) and colorectal cancers (13%), had a high number of risk factors and diverse and unmeasured exposure patterns among groups, likely reflecting considerable genetic susceptibilities.

The article "Causes of Cancer in the World: Comparative Risk Assessment of Nine Behavioral and Environmental Risk Factors" was retracted in 2024. Reasons: plagiarism; plagiarized images; overlap with other authors' work.

Lung cancer accounted for 37% of all risk factor-related mortality, liver cancer accounted for 11%, and esophageal cancer accounted for 27% (271,000 deaths), showing that significant numbers of cancer-related deaths were aﬀected by the union of relatively large joint PAFs (Table 2). Patients with three malignancies have a five-year survival rate of <25%. Leukemia and corpus uteri cancer were the two illnesses that caused the least fatalities (23,000 and 28,000, respectively). As it was challenging to convert exposure to new geographies, the 3% of leukemia fatalities linked to professional exposures were not reanalyzed and were not included in this study.

Despite only possessing 15% of the global population, high-income nations were responsible for 30% of the 7,000,000 cancer mortality worldwide and 31% of the 243 million fatalities that may be attributed to the dangers indicated in Table 1 (21% of those under the age of 30). In middle- and low-income countries, there were another 17% of attributable fatalities. All cancer sites reported larger combined PAFs in high-income nations than in the middle- and low-income ones, except for cervix uteri cancer. This finding, particularly pronounced for cancers of the mouth, oropharynx, and esophagus, as well as esophageal malignancies, especially in men, is mostly due to longer and higher community exposure to alcohol consumption and smoking. However, for both countries, the total PAFs for all malignancies were comparable. There is a smaller diﬀerence between PAFs for all sites and PAFs for those cancers because various site-specific cancer subtypes contribute diﬀerently to overall cancer mortality. Additionally, these cancer sites were the cause of 25% of cancer mortality in high-income countries but only 18% of cancer deaths overall in middle- and low-income countries.

In middle- and low-income nations, the majority of fatalities were caused by lung, liver, and esophageal cancers. Lung cancer accounted for 396,000 (52%) of all cancer mortality in high-income countries; the remaining 72% of cancer fatalities were due to other malignancies. This shows the effectiveness of some preventive measures as well as the disproportionate growth in lung cancer deaths in many high-income countries where smoking incidence is still high.

Europe and Central Asia (ECA), which had the greatest joint PAF for all cancer sites combined in low- and middle-income nations, had a 39% rate, whereas sub-Saharan Africa (SSA), as well as North Africa and the Middle East (MENA), had the lowest joint PAF at 24% (MENA; 24%). ECA had the highest joint PAF among men (50%) and the lowest joint PAF among SSA (19%), with smoking, drinking, being overweight, and obesity having a big influence on both. SSA had the greatest combined PAF for women (29%), while MENA had the lowest (19%). The high mortality rate from cervix uteri cancer, which is significantly impacted by the lack of access to cervical screening and the sexual transmission of HPV, was a major contributor to the high PAF for women in SSA.

The article "Causes of Cancer in the World: Comparative Risk Assessment of Nine Behavioral and Environmental Risk Factors" was retracted in 2024. Reasons: plagiarism; plagiarized images; overlap with other authors' work.

The majority of fatalities in low- and middle-income countries that could be attributed to the hazards listed in Table 1 were found in EAP (746,000; 45% of all cancer deaths that could be attributed in low- and middle-income countries), ECA (324,000; 19%), and South Asia (SAR: 322,000; 19%). The overall number of cancer-related fatalities is high in all three areas, mostly due to the dense populations in EAP and SAR. Although fewer people are living in ECA, there are still a lot of people dying from cancer overall, and a greater percentage of those deaths are caused by these risk factors individually and together, particularly smoking.

MENA and SSA had the lowest cancer fatalities that might be directly associated with the risk variables we studied due to the lower overall number of cancer mortality and the lower PAFs resulting from these hazards.

According to estimates, smoking alone is responsible for 21% of cancer mortality globally. Another 5% was caused by drinking and having inadequate amounts of fruits and vegetables. Due to shorter smoking history and a lower incidence among women, smoking caused a huge percentage of cancer mortality in high-income nations (29%) compared to middle- and low-income regions (18%). However, due to the higher overall number of cancer mortality in middle- and low-income countries (896,000 versus 596,000), the number of smoking-related cancer fatalities was higher. Because there were so many fatalities in ECA and EAP that might be attributed to alcohol consumption, the all-cancer-site PAF for alcohol use was comparable in the two regions. The most fatalities from alcohol-related causes in EAP were related to cancers of the liver and esophagus.

Smoking and alcohol use are hazards with proven treatments that have considerably increased cancer deaths in middle- and low-income regions. In hospital settings, contaminated injections caused 108,000 fatalities throughout the six regions, with EAP accounting for 91,000 of those fatalities. In total, 16,000 lung cancer fatalities were caused by indoor smoke from solid fuels, which was exclusively an issue in the EAP and SAR regions where coal is utilized [30].

The article "Causes of Cancer in the World: Comparative Risk Assessment of Nine Behavioral and Environmental Risk Factors" was retracted in 2024. Reasons: plagiarism; plagiarized images; overlap with other authors' work.

Obesity and inactivity were the leading causes of all-site cancer deaths in ECA, showing that this group was significantly exposed to these lifestyle-related risk factors, which coexist with the risk from smoking and alcohol use. The risk variables included in this study contributed to 41% of cancer deaths in men compared to 27% in women, or almost two times as much cancer mortality in men as in women. For males, lung cancer accounted for 45% of all fatalities attributed to risk factors, and for women, cervix uteri cancer (28% of all attributable deaths). Diﬀerences in PAFs and attributable fatalities between men and women were significantly influenced by smoking and alcohol use. Except for cervix, corpus uteri, and breast cancers and their specific risk factors, which virtually exclusively impact women, the total number of fatalities from major cancers and the number attributed to the primary hazards were higher in men than in women (Figure 2). For colon cancer, where it is unknown whether smoking or drinking alcohol significantly aﬀects risk, this pattern did not remain true. Alcohol and smoking had a considerable influence on the risk of developing oral or oropharynx cancer, and PAFs for this disease revealed the highest gender gap (23% for women vs. 66% for men). In middle- and low-income countries, mouth or oropharynx cancer also had the highest gender difference (17% for women vs. 63% for men), whereas liver cancer had one of the highest gender differences in high-income nations. The age group of 30-69 years had the biggest combined PAFs, except for lung cancer in high-income countries. Cohort eﬀects of exposure to alcohol usage and smoking contributed to this. Between the ages of 30 and 69, cancer fatalities accounted for more than half of all deaths (Table 3). This age group also had the highest incidence of cancer-related fatalities, except bladder cancer, which suggests that lowering exposure to these risk factors might result in a significant increase in life expectancy. The most cancer-related fatalities in the youngest age group (under 30 years) were caused by leukemia. None of the leukemia fatalities at these ages was associated with the risk factors we examined, which is surprising given that most epidemiological studies only assess risks after 30 years of age. The eﬀectiveness of the cancer prevention programs for young people in high-income countries is demonstrated by the fact that middle- and low-income countries had significantly higher PAFs and noticeably higher death rates in this age group, even though the overall number of cancer-related deaths among people under 30 was generally low.

The article "Causes of Cancer in the World: Comparative Risk Assessment of Nine Behavioral and Environmental Risk Factors" was retracted in 2024. Reasons: plagiarism; plagiarized images; overlap with other authors' work.

Discussion

Nine potentially modifiable risk factors account for more than one in three of the 7 million cancer-related deaths globally, with drinking and smoking contributing significantly in both low-and high-income countries. A significant risk component for women is the sexual transmission of HPV, which can result in chronic infection and the spread of cancer-causing virus strains. This is especially true in the poorest regions where access to cervical cancer screening is scarce. This fraction may significantly rise for different cancer regions depending on other potentially modifiable risk variables not mentioned here. Doll and Peto’s [18] estimate, which was based on a comparison of age-standardized incidence rates from the United States from 1978 with the lowest reliably documented incidence rates in other populations, accounts for nearly half of our estimate of the percentage of fatalities globally attributable to the nine risk variables we evaluated. Because Doll and Peto [18] compared incidence rates, their predictions account for changes in exposure to all known and unknown risk factors.

Additionally, just the United States was included in their calculations. Consequently, there is no direct comparison between Doll and Peto’s estimates and ours. Some significant malignancies, such as kidney, prostate, lymphomas, and melanoma, were not linked to any of these risks we examined. These malignancies have several known or improbable behavioral and environmental hazards, as well as varied exposure patterns that make it challenging to quantify exposure and risk. Additionally, we did not evaluate several well-known risk variables, including professional exposure, which caused 102,000 cancer mortality worldwide, exposure to *Helicobacter pylori* in food, UV radiation exposure, and ambient cigarette smoke. Due to the diﬃculties in obtaining accurate exposure estimates from available data, we mostly disregarded these factors from our analysis.

Our estimates are subject to several sources of uncertainty, particularly those that entail extrapolating exposure and risk from one group to another. The explanations about the data sources of each risk factor go into further depth [21-31]. There have also been other descriptions of the origins of uncertainty in the assumptions and methodologies used to estimate joint PAFs and the sensitivity of the results to these assumptions [32]. In addition to the individual and combined PAFs, the total site-specific cancer mortality to which the PAFs are applied is unknown [33,34]. There are around 75 nations with relatively full vital records and death certifications [33,34]. Another 51 countries employ sample registration or surveillance methods or have inadequate vital statistics. The 65 remaining nations, most of which are in SSA, lack accurate information on adult mortality. For these populations, the WHO estimates the age-specific all-cause mortality rates using conventional demographic techniques [35]. The overall number of cancer deaths is estimated for nations with limited data using cause-of-death models. Regional incidence or death trends from cancer registries, which submit data to the IARC [36], or cancer survival models without such information, are used to determine the distribution of cancer fatalities by the site. For most WHO member nations, IARC also oﬀers estimates of location-wise cancer mortality. The ramifications of these various techniques have already been examined, along with a comparison of them [33,34]. Consequently, with bigger discrepancies for SSA, SAR, and MENA, worldwide cancer mortality estimates provided by the WHO are 11% higher than those offered by the IARC.

The article "Causes of Cancer in the World: Comparative Risk Assessment of Nine Behavioral and Environmental Risk Factors" was retracted in 2024. Reasons: plagiarism; plagiarized images; overlap with other authors' work.

In affluent countries, decades of biomedical research have produced several successful therapies that reduce the incidence and mortality of cancer. Examples include the hepatitis B vaccine for liver cancer, screening methods for cervical cancer [37,38], fecal occult blood test for colorectal cancer [39-41], mammography for breast cancer [42,43], hepatitis B vaccine for liver cancer, the surgical prevention of colorectal cancers, and others [44]. Increased use of the technologies mentioned above, particularly those that require early diagnosis, would undoubtedly contribute to further lowering the burden of cancer. Less progress has been made in the fight against other cancers, chest X-rays and sputum cytology for lung cancer have not been encouraging, and vaccines for HPV and *H. pylori* are currently being researched [45,46]. The eﬀectiveness of radiation and chemotherapy diﬀer from cancer to cancer and is influenced by various biological and technological parameters, including the stage of the disease.

## Conclusions

The fixation on healing advanced diseases has hampered the fight against cancer. Additionally, the accessibility and uptake of preventative, screening, and treatment interventions, factors that heavily depend on the cost and the characteristics of the health system, will only impact population statistics if implemented. These obstacles prevent these therapies from being used widely in places with limited resources. These limitations highlight the significance of our findings for programs and policies that alter social and environmental conditions to reduce cancer incidence.
